RETRACTED

# Kaempferol suppresses human gastric cancer SNU-216 cell proliferation, promotes cell autophagy, but has no influence on cell apoptosis

**DOI:** 10.1590/1414-431X20187843

**Published:** 2019-02-14

**Authors:** Fan Zhang, Cuimei Ma

**Affiliations:** 1 Teaching and Research Department of Diagnostics, Jining Medical University, Jining, China; 2 Department of Gastroenterology, Affiliated Hospital of Jining Medical University, Jining, China

**Keywords:** Gastric cancer, Kaempferol, MicroRNA-181a, Cell proliferation, Cell autophagy

## Abstract

Gastric cancer remains a serious threat to human health worldwide. Kaempferol is a plant-derived flavonoid compound with a wide range of pharmacological activities. This study aimed to investigate the effects of kaempferol on gastric cancer SNU-216 cell proliferation, apoptosis, and autophagy, as well as underlying potential mechanisms. Viability, proliferation, and apoptosis of SNU-216 cells after kaempferol treatment were evaluated using cell counting kit-8 assay, 5-btomo-2′-deoxyuridine incorporation assay, and annexin V-FITC/PI staining, respectively. Quantitative reverse transcription PCR was performed to measure the mRNA expressions of cyclin D1 and microRNA-181a (miR-181a) in SNU-216 cells. Cell transfection was used to down-regulate the expression of miR-181a. The protein expression levels of cyclin D1, bcl-2, bax, caspase 3, caspase 9, autophagy-related gene 7, microtubule-associated protein 1 light chain 3-I (LC3-I), LC3-II, Beclin 1, p62, mitogen-activated protein kinase (MAPK), extracellular regulated protein kinases (ERK), and phosphatidylinositol 3 kinase (PI3K) in SNU-216 cells were detected using western blotting. Results showed that kaempferol significantly suppressed SNU-216 cell viability and proliferation but had no influence on cell apoptosis. Further results suggested that kaempferol significantly induced SNU-216 cell autophagy. The expression of miR-181a in SNU-216 cells after kaempferol treatment was enhanced. Kaempferol significantly inactivated MAPK/ERK and PI3K pathways in SNU-216 cells. Suppression of miR-181a significantly reversed the kaempferol-induced MAPK/ERK and PI3K pathways inactivation in SNU-216 cells. This research demonstrated that kaempferol suppressed proliferation and promoted autophagy of human gastric cancer SNU-216 cells by up-regulating miR-181a and inactivating MAPK/ERK and PI3K pathways.

## Introduction

Gastric cancer is a major health burden worldwide, which accounts for roughly 28,000 new cases and 10,960 deaths per year (1,2). According to the results of epidemiology research, multiple factors contribute to the occurrence of gastric cancer, including improper dietary habits and life style, *Helicobacter pylori* infection, and chronic stomach disease (3,4). Although diagnosis and treatment of gastric cancer have improved in recent years, the 5-year survival rate of patients remains only 30% (5). The lack of effective early diagnostic biomarkers and the side effects of systemic therapies are major reasons for death (6,7). Therefore, searching for novel and more effective preventive, diagnostic, and therapeutic strategies for gastric cancer are still extremely needed.

RETRACTED

Plant-derived medicines in cancer therapy have gained more attention around the world, due to their safety, efficiency, and minimal side effects (8). Kaempferol is a natural flavonoid compound found in many vegetables and fruits with a wide range of pharmacological activities (9,10). Regarding its anti-cancer effects, several preliminary studies demonstrated that kaempferol suppressed the growth of multiple cancers, including breast cancer (11), lung cancer (12), colon cancer (13), bladder cancer (14), hepatic cancer (15), pancreatic cancer (16), and gastric cancer (17). For gastric cancer, Song et al. (17) demonstrated that kaempferol suppressed the proliferation of human gastric cancer MKN28 and SGC7901 cells, as well as the growth of tumor xenografts, by inactivating phosphatidylinositol 3 kinase/protein kinase 3 (PI3K/AKT) and mitogen-activated protein kinase/extracellular regulated protein kinases (MAPK/ERK) signaling pathways. More experimental research is still needed to further explore the specific molecular mechanisms of kaempferol on gastric cancer cells.

MicroRNAs (miRNAs) are small non-coding regulatory RNAs in eukaryotic cells, which can serve as gene regulators capable of controlling expression of multiple genes by targeting the 3′ untranslated regions (3′UTR) of the mRNAs (18). Kaempferol can exert anti-cancer effects by regulating miRNAs expressions in cancer cells (19). Previous experimental study showed that miRNA-181a (miR-181a) was down-regulated in gastric cancer tissues and played critical roles in suppressing gastric cancer HGC-27 cell proliferation, invasion, and metastasis (20). However, there is no information available about the effects of kaempferol on miR-181a expression in gastric cancer cells.

Thus, in this research, we assessed the proliferation, apoptosis, and autophagy of human gastric cancer SNU-216 cells after kaempferol treatment. Moreover, we analyzed the role of miR-181a in kaempferol-induced inactivation of MAPK/ERK and PI3K pathways in SNU-216 cells. These findings will provide new evidence for further understanding the anti-cancer effects of kaempferol on gastric cancer.

## Material and Methods

### Cell culture and treatment

Human gastric cancer cell line SNU-216 was provided by Korean Cell Line Bank (Korea). Human gastric epithelial GES-1 cells were purchased from Beijing Institute for Cancer Research (China). SNU-216 and GES-1 cells were both cultured in Dulbecco’s modified Eagle’s medium (DMEM, Sigma-Aldrich, USA) supplemented with 10% fetal bovine serum (FBS, Gibco, Life Technologies, USA), 1% penicillin-streptomycin (Gibco, Life Technologies), and 1 mM L-glutamine (Sigma-Aldrich, USA). Cultures were maintained in a humidified incubator (Thermo Fisher Scientific, USA) at 37°C with 5% CO_2_.

RETRACTED

Kaempferol powder was obtained from Sigma-Aldrich (catalog number: K0133, USA) and dissolved in dimethyl sulfoxide (DMSO, Thermo Fisher Scientific) to a final storage concentration of 100 mM according to the manufacturer’s instruction. Serum-free DMEM was used to dilute kaempferol solution to 10–100 μM before experiments. The chemical structure of kaempferol is displayed in Figure 1.

**Figure 1.** The chemical structure of kaempferol.

### Cell viability assay

Cell viability was measured using cell counting kit-8 (CCK-8, Beyotime Biotechnology, China) assay. Briefly, GES-1 or SNU-216 cells were seeded in a 96-well plate (Costar, Corning Incorporated, USA) with 1 × 10^4^ cells per well and exposure to 10–100 μM kaempferol for 24 or 48 h. Then, 10 μL CCK-8 solution was added into each well of the plate followed by incubation for 1 h at 37°C. After that, the absorbance of each well at 450 nm was recorded using a micro-plate reader (Bio-Tek Instruments, USA). Cell viability (%) was quantified by average absorbance of kaempferol treatment group/average absorbance of control group × 100%.

### Cell proliferation assay

Cell proliferation was evaluated using 5-bromo-2′-deoxyuridine (BrdU) incorporation assay (Calbiochem, USA) according to the manufacturer’s protocol. Briefly, SNU-216 cells were seeded in 6-well plates (Costar, Corning Incorporated) with 1 × 10^5^ cells per well. BrdU (1 mg/mL) was added into each well of the plate before 50 μM kaempferol treatment for 4 h. Incubation time with kaempferol was 24 h. After that, cell proliferation (%) of each group was quantified by number of BrdU positive (+) cells/number of total cells × 100%.

### Quantitative reverse transcription PCR (qRT-PCR)

qRT-PCR was conducted to detect the expressions of cyclin D1 and miR-181a in SNU-216 cells after 50 μM kaempferol treatment or miR-181a inhibitor transfection. Briefly, after relevant treatment or transfection, total RNAs in SNU-216 cells were isolated using TRIzol^TM^ Plus RNA Purification kit (Invitrogen, USA). SuperScript^TM^ III Platinum^TM^ One-Step qRT-PCR kit (Invitrogen) was used to detect the expressions of cyclin D1 and β-actin. MirVana^TM^ qRT-PCR miRNA Detection kit (Invitrogen) was used to detect the expression of miR-181a and U6; β-actin and U6 acted as endogenous control, respectively. The primers were cyclin D1: 5′-CCCTCGGTGTCCTACTTCAAA-3′ (forward) and 5′-CACCTCCTCCTCCTCCTCTTC-3′ (reverse); β-actin: 5′-CCAGGCACCAGGGCGTGATG-3′ (forward) and 5′-CGGCCAGCCAGGTCCAGACG-3′ (reverse); miR-181a: 5′-GAACATTCAACGCTGTCGGTG-3′; U6: 5′-TGCGGGTGCTCGCRRCGGCAGC-3′. Data was quantified using 2^−△△Ct^ method (21).

RETRACTED

### Cell apoptosis assay

Cell apoptosis was determined using annexin V-FITC/PI apoptosis detection kit (Becton-Dickinson, USA) following the manufacturer’s instructions. SNU-216 cells were seeded in a 6-well plate (Costar, Corning Incorporated) with 1 × 10^5^ cells per well and exposure to 50 μM kaempferol for 24 h. Then, cells in each well were harvested, washed twice with phosphate buffered saline (PBS, Beyotime Biotechnology), and stained with annexin V-FITC/PI solution for 25 min at 37°C in the dark. FACScan flow cytometry (BD Biosciences, USA) was performed to analyze cell apoptosis. Data were quantified using FlowJo software (FlowJo LLC, USA) (22).

### Cell transfection

miR-181a inhibitor and negative control (NC) were both designed and synthesized by GenePharma Corporation (China). The sequence for miR-181a inhibitor was: 5′-ACUCACCGACAGCGUUGAAUGUU-3′. Cell transfection was conducted using Lipofectamine 3000 reagent (Invitrogen) in line with the manufacturer’s protocol. Transfection efficiency was evaluated using qRT-PCR.

### Western blotting

After 50 μM kaempferol treatment and/or miR-181a inhibitor transfection, total proteins in SNU-216 cells were isolated using RIPA lysis and extraction buffer (Thermo Fisher Scientific, USA) and quantified using BCA protein assay kit (Beyotime Biotechnology). Bio-Rad Bis-Tris Gel system (Bio-Rad Laboratories, USA) was used to establish the western blotting system. Then, proteins in equal concentrations were electrophoresed in polyacrylamide gels and transferred onto nitrocellulose membranes (Millipore, USA), which were incubated with primary antibodies. All primary antibodies were prepared in 1% bovine serum albumin (BSA, Beyotime Biotechnology) solution at a dilution of 1:1000. Anti-cyclin D1 antibody (#2922), anti-Bcl-2 antibody (#2872), anti-Bax antibody (#2774), anti-pro-caspase 3 antibody (#9662), anti-cleaved-caspase 3 antibody (#9664), anti-pro-caspase 9 antibody (#9502), anti-cleaved-caspase 9 antibody (#9505), anti-autophagy-related gene 7 (ATG7) antibody (#2631), anti-microtubule-associated protein 1 light chain 3-I/II (LC3-I/II) antibody (#4108), anti-beclin 1 antibody (#3738), anti-p62 antibody (#8025), anti-MAPK antibody (#9212), anti-p-MAPK antibody (#9216), anti-ERK antibody (#9102), anti-p-ERK antibody (#5726), anti-PI3K antibody (#4292), anti-p-PI3K antibody (#4228), and anti-β-actin antibody (#4970) were all purchased from Cell Signaling Technology (USA). Subsequently, the nitrocellulose membranes were incubated with anti-mouse (rabbit) IgG (H+L) DYLight^TM^ 680 conjugate (#5470, #5366, Cell Signaling Technology) for 1 h at room temperature. Odyssey System (Licor Biosciences, Germany) was used to record signals of proteins. Data were quantified using Quantity One software (Bio-Rad Laboratories) (23).

RETRACTED

### Statistical analysis

All experiments were repeated at least three times. GraphPad 6.0 software (GraphPad, USA) was used for statistical analysis. Data are reported as means±SD. Statistical comparisons were made using Student’s *t*-test or one-way analysis of variance (ANOVA). P<0.05 was considered statistically significant.

## Results

### Kaempferol suppressed SNU-216 cell viability and proliferation

Firstly, we detected the viability of GES-1 cells after 10–100 μM kaempferol treatment using CCK-8 assay. Results in Figure 2A show that 10–50 μM kaempferol treatment had no significant effect on GES-1 cell viability, while 60-100 μM kaempferol treatment inhibited the viability of GES-1 cells (P<0.05 or P<0.01). These results suggested that high concentrations of kaempferol (over 50 μM) might have toxic effects on human normal gastric cells. The viability of SNU-216 cells after 10–50 μM kaempferol treatment for 24 and 48 h were then measured. Figure 2B and C show that kaempferol inhibited the viability of SNU-216 cells in a dose- and time-dependent manner (P<0.05 or P<0.01). Kaempferol treatment at 50 μM for 24 h reduced the viability of SNU-216 cells to 26.87±3.18% and 50 μM kaempferol treatment for 48 h reduced the viability of SNU-216 cells to 9.63±4.28%. Considering that 50 μM kaempferol treatment for 24 h was able to significantly inhibit the viability of SNU-216 cells, this protocol was chosen for subsequent experiments. Figure 2D displays that, compared to the control group, the rate of BrdU positive (+) cells in 50 μM kaempferol treatment group was significantly reduced (P<0.01). In addition, qRT-PCR and western blotting illustrated that the mRNA and protein expression levels of cyclin D1 in SNU-216 cells were both decreased after 50 μM kaempferol treatment (Figure 2E and F, P<0.01). The above results indicated that appropriate concentration of kaempferol could suppress gastric cancer SNU-216 cell viability and proliferation, but had no significant effect on normal gastric cells.

RETRACTED

**Figure 2.** Kaempferol suppressed SNU-216 cell viability and proliferation. *A*, Viability of GES-1 cells after 10–100 μM kaempferol treatment was detected using cell counting kit-8 assay. *B* and *C*, Viability of SNU-216 cells after 10–50 μM kaempferol treatment for 24 and 48 h were measured using CCK-8 assay. *D*, Proliferation of SNU-216 cells after 50 μM kaempferol treatment was evaluated using 5-bromo-2′-deoxyuridine incorporation assay (BrdU). *E* and *F*, mRNA and protein expression levels of cyclin D1 in SNU-216 cells after 50 μM kaempferol treatment were determined using quantitative reverse transcription PCR and western blotting, respectively. Data are reported as means±SD. *P<0.05, **P<0.01 (ANOVA or *t*-test).

### Kaempferol had no influence on SNU-216 cell apoptosis

Annexin V-FITC/PI staining and western blotting were performed to assess SNU-216 cell apoptosis after 50 μM kaempferol treatment for 24 h. As displayed in Figure 3A, the rate of apoptotic cells was not changed after 50 μM kaempferol treatment, compared to the control group. The expression levels of bcl-2, bax, pro-capsase 3, cleaved-caspase 3, pro-caspase 9, and cleaved-caspase 9 were also not changed in SNU-216 cells after 50 μM kaempferol treatment, compared to the control group (Figure 3B). These findings suggested that kaempferol had no influence on SNU-216 cell apoptosis.

**Figure 3.** Kaempferol had no influence on SNU-216 cell apoptosis. *A*, Annexin V-FITC/PI staining was used to assess the apoptosis of SNU-216 cells after 50 μM kaempferol treatment. *B*, Western blotting was performed to detect the expressions of Bcl-2, Bax, pro-caspase 3, cleaved-caspase 3, pro-caspase 9, and cleaved-caspase 9 in SNU-216 cells after 50 μM kaempferol treatment. Data are reported as means±SD (*t*-test).

### Kaempferol induced SNU-216 cell autophagy

To analyze the effects of kaempferol on SNU-216 cell autophagy, the protein expression levels of ATG7, LC3-I, LC3-II, beclin 1, and p62 in SNU-216 cells after 50 μM kaempferol treatment were measured using western blotting. Figure 4A and B show that 50 μM kaempferol treatment significantly down-regulated the protein expression level of p62 (P<0.01) and remarkably up-regulated the protein expression levels of ATG7, LC3-II/I, and beclin 1 in SNU-216 cells (P<0.05 or P<0.01). These findings revealed that kaempferol obviously induced gastric cancer SNU-216 cell autophagy.

**Figure 4.** Kaempferol induced SNU-216 cell autophagy. After 50 μM kaempferol treatment, the protein expression levels of ATG7, LC3-I, LC3-II, beclin 1, and p62 in SNU-216 cells were evaluated using western blotting. ATG7: autophagy-related gene 7; LC3: microtubule-associated protein 1 light chain 3. Data are reported as means±SD. *P<0.05, **P<0.01 (*t*-test).

RETRACTED

### Kaempferol up-regulated the expression of miR-181a in SNU-216 cells

The expression level of miR-181a in SNU-216 cells after kaempferol treatment was detected using qRT-PCR. Results in Figure 5 show that 50 μM kaempferol treatment significantly enhanced the expression level of miR-181a in SNU-216 cells (P<0.01). This result implied that miR-181a might participate in the effects of kaempferol on SNU-216 cell proliferation, inhibition, and autophagy occurrence.

**Figure 5.** Kaempferol up-regulated the expression of microRNA (miR)-181a in SNU-216 cells. Quantitative reverse transcription PCR was conducted to determine the expression of miR-181a in SNU-216 cells after 50 μM kaempferol treatment. Data are reported as means±SD. **P<0.01 (*t*-test).

### Kaempferol inactivated MAPK/ERK and PI3K pathways in SNU-216 cells

The activation of MAPK/ERK and PI3K in SNU-216 cells after kaempferol treatment was evaluated using western blotting. As displayed in Figure 6, 50 μM kaempferol treatment significantly reduced the expression rates of p-MAPK/MAPK, p-ERK/ERK, and p-PI3K/PI3K in SNU-216 cells (P<0.01). These findings indicated that kaempferol could inactivate MAPK/ERK and PI3K pathways in gastric cancer SNU-216 cells.

**Figure 6.** Kaempferol inactivated MAPK/ERK and PI3K pathways in SNU-216 cells. After 50 μM kaempferol treatment, the expressions of MAPK, p-MAPK, ERK, p-ERK, PI3K, and p-PI3K in SNU-216 cells were determined using western blotting. MAPK: mitogen-activated protein kinase; ERK: extracellular regulated protein kinases; PI3K: phosphatidylinositol 3 kinase. Data are reported as means±SD. **P<0.01 (*t*-test).

### miR-181a participated in the kaempferol-induced MAPK/ERK and PI3K pathways inactivation in SNU-216 cells.

Finally, to verify the roles of miR-181a in kaempferol-induced MAPK/ERK and PI3K pathways inactivation, miR-181a inhibitor was transfected into SNU-216 cells. Results in Figure 7A illustrate that miR-181a inhibitor transfection significantly down-regulated the expression level of miR-181a in SNU-216 cells (P<0.01). Figure 7B shows that miR-181a inhibitor transfection notably reversed the kaempferol-induced MAPK/ERK and PI3K pathways inactivation in SNU-216 cells by enhancing the expression rates of p-MAPK/MAPK, p-ERK/ERK and p-PI3K/PI3K (P<0.01). These findings suggested that miR-181a played critical roles in kaempferol-induced MAPK/ERK and PI3K pathways inactivation in gastric cancer SNU-216 cells.

**Figure 7.** microRNA (miR)-181a participated in the kaempferol-induced MAPK/ERK and PI3K pathways inactivation in SNU-216 cells. *A*, After miR-181a inhibitor transfection, the expression of miR-181a in SNU-216 cells was detected using quantitative reverse transcription PCR. *B*, Western blotting was performed to evaluate the expressions of MAPK, p-MAPK, ERK, p-ERK, PI3K, and p-PI3K in SNU-216 cells after 50 μM kaempferol treatment and/or miR-181a inhibitor transfection. NC: negative control; MAPK: mitogen-activated protein kinase; ERK: extracellular regulated protein kinases; PI3K: phosphatidylinositol 3 kinase. Data are reported as means±SD.**P<0.01 (ANOVA).

RETRACTED

## Discussion

As one of the most common gastrointestinal tumors, gastric cancer remains a serious threat to human health worldwide (1,24). In this research, we showed that kaempferol, a plant-derived flavonoid compound, inhibited gastric cancer SNU-216 cell proliferation and induced cell autophagy. Moreover, kaempferol enhanced the expression of miR-181a in SNU-216 cells. Furthermore, miR-181a participated in the kaempferol-induced inactivation of MAPK/ERK and PI3K pathways in SNU-216 cells.

Plant-derived medicines have made their own niche in the treatment of multiple diseases, including cancers (25,26). An epidemiology study demonstrated that there was a negative association between occurrences of cancers and consumption of foods containing kaempferol (27). In this study, we found that an appropriate concentration of kaempferol could reduce gastric cancer SNU-216 cell viability and proliferation, but had no influence on cell apoptosis. The mRNA and protein expression levels of cyclin D1, which plays pivotal roles in cancer cell proliferation (28), were both decreased after kaempferol treatment. Considering that kaempferol had been found to exert anti-proliferative effects on gastric cancer MKN28 and SGC7901 cells (17), the results of our research further indicated that kaempferol could suppress multiple gastric cancer cell proliferation.

Cell autophagy has been considered as a non-apoptotic form of programmed cell death (29). Guo et al. (30) suggested that kaempferol induced hepatic cancer cell death through endoplasmic reticulum stress-CCAAT/enhancer-binding protein homologous protein (CHOP)-autophagy signaling pathway. Huang et al. (15) proved that kaempferol induced human hepatic cancer cell autophagy via adenosine 5′-monophosphate-associated protein kinase (AMPK) and AKT signaling pathways. Thus, in the present research, we also investigated the effects of kaempferol on gastric cancer SNU-216 cell autophagy. We found that the protein expression levels of ATG7, LC3-II/I, and beclin 1 were all enhanced and the protein expression level of p62 was decreased in SNU-216 cells after kaempferol treatment. ATG7 is a core autophagy regulator and required for autophagy-dependent lipid metabolism (31). During autophagy, a cytosolic form of LC3 (LC3-I) is lapidated and converted to form LC3-II, which is a key process of autophagy pathway (32). Beclin 1 is a positive regulator of cell autophagy and p62 is a negative regulator of cell autophagy (33,34). Therefore, we could conclude that kaempferol also played anti-cancer effects on gastric cancers by inducing gastric cancer cell autophagy.

RETRACTED

Numerous studies demonstrated that miRNAs had critical roles in the regulation of multiple cellular processes and participated in the progression of many cancers (35). Many plant-derived medicines, including kaempferol, can exert anti-cancer effects by modulating the expressions of miRNAs (19,36). In this research, we revealed that kaempferol enhanced the expression level of miR-181a in SNU-216 cells, suggesting that miR-181a might participate in the effects of kaempferol on gastric cancer cells. Moreover, this result was consistent with a previous study, which showed that miR-181a was down-regulated in gastric cancer tissues and played central roles in suppressing gastric cancer HGC-27 cell proliferation, invasion, and metastasis (20).

Song et al. (17) reported that kaempferol suppressed the proliferation of gastric cancer cells by inactivating PI3K/AKT and MAPK/ERK signaling pathways. Consistent with this previous study, we also found that kaempferol could inactivate MAPK/ERK and PI3K pathways in gastric cancer SNU-216 cells. Moreover, suppression of miR-181a reversed the kaempferol-induced MAPK/ERK and PI3K pathways inactivation in SNU-216 cells. These findings suggested that miR-181a participated in the kaempferol-induced inactivation of MAPK/ERK and PI3K pathways in gastric cancer SNU-216 cells. Considering that MAPK/ERK and PI3K pathways played critical roles in promoting gastric cancer cell proliferation and autophagy (37,38), the results of our research implied that kaempferol suppressed gastric cancer cell growth by up-regulating miR-181a and inactivating MAPK/ERK and PI3K pathways.

In conclusion, our research demonstrated that kaempferol suppressed proliferation and promoted autophagy of human gastric cancer SNU-216 cells by up-regulating miR-181a and inactivating MAPK/ERK and PI3K pathways. This study will be helpful for further understanding the anti-cancer effects of kaempferol on gastric cancer and provide a theoretical basis for deeply exploring the treatment of gastric cancer by kaempferol.
